This article has been retracted.

# Analysis of Teaching Strategies of College English Speculative Reading Based on Big Data Analysis of Student Behavior in Cross-Cultural Education Environment

**DOI:** 10.1155/2022/1385074

**Published:** 2022-09-10

**Authors:** Nannan Du

**Affiliations:** Department of Foundational Courses, Nanjing Vocational University of Industry Technology, Nanjing 210023, China

## Abstract

Both dynamic and interactive, cross-cultural education emphasizes respect, interaction, and understanding between various cultural groups. Its fundamental principle is to acknowledge and value cultural diversity while opposing attempts to artificially unite cultures in order to recognise the equality and common heritage of all cultures. The goal of intercultural education, from an individual's perspective, is to support those who are educated in understanding, accepting, and respecting other foreign cultures in order to better adapt to and thrive in a multicultural society. To develop students' intercultural communication skills is the goal of intercultural education. Based on the associations between intercultural education and speculative reading, this essay analyzes the crucial role that intercultural English teaching and speculative reading instruction play in colleges and universities before going over the situation and approaches that English speculative reading instruction is currently facing. This paper primarily discusses the data on students from the student work management system, the relationship between grades and actual behavior, and the rules that are mined to provide a scientific basis for decision-making for the relevant units in colleges and universities. According to experimental analysis, the data mining algorithm in this paper performs better than the other two in terms of predicting students' English achievement, with an average accuracy of 0.86 compared to 0.71, 0.075, and 0.73 for the other three algorithms. The decision tree created using this methodology can quantitatively reflect the impact of different teaching factors on learning quality and offers a clear and reliable foundation for formulating targeted improvement strategies.

## 1. Introduction

The demand gap for international talent has been growing over the past few years as a result of the rapid development of economic globalisation, which has raised the bar for the education and instruction provided by colleges and universities in order to develop talent from abroad. In order to develop students' English language proficiency, college English—an essential component of the college curriculum system—should be combined with the demands of international talent training in teaching practice, with an emphasis on developing students' intercultural communication and critical thinking skills in English [1]. The teaching strategy of instilling theoretical knowledge, such as words and grammar, has long been used in the teaching practice of speculative reading in college English. As a result, college students have become popular products in modern educational production, severely lacking the ability to engage in critical thought and engage in cross-cultural communication, and unable to meet the actual needs of economic globalisation [2, 3]. This led to the creation of the teaching of English speculative reading based on cross-cultural education, which was then popularised and applied in the teaching and practice of English speculative reading in colleges and universities, providing a guarantee for developing global talents. Reading is a key way for students to learn a language, and colleges and universities are the birthplace of developing high-quality English talents [4]. Thinking across cultures, teaching students to read in English is a crucial step in developing their proficiency in the language as well as their intercultural, cognitive, and humanistic qualities. The original English teaching method of speculative reading is no longer able to meet the demands of social development due to the advancement of global integration. Teachers should adapt to the new era, define the meaning of cross-cultural speculative reading teaching, comprehend its significant value, and develop scientific teaching strategies that are tightly centred around the core teaching content.

Speculative reading refers to an effective way for readers to make full use of multiple means, such as explanation and inference, to deeply understand the connotation of an article. Speculative reading emphasizes that reading is an effective means. However, in the process of reading an article, readers should not stay at the simple mastery of words and the understanding of the superficial meaning of sentences but should thoroughly study the author's true feelings and intentions in writing, so as to guess the connotation contained in the article on the basis of objectively evaluating the author's views, and then dialectically and creatively understand the connotation of the article, and finally form personalized opinions. On the basis of cultivating students' language ability, cross-cultural critical reading teaching highlights the cultivation of cross-cultural ability and critical ability, which is conducive to improving students' comprehensive quality. Reading can not only consolidate students' basic language skills but also cultivate students' thinking ability and analytical ability, making them a high-quality English professional [5]. Cross-cultural competence refers to students' ability to accept, understand, and apply the cultures of English-speaking countries. Cross-cultural communication is a very important part of college English humanistic quality education. It can cultivate and improve English majors' cross-cultural communication ability, cultivate their cross-cultural sensitivity and consciousness, and enable students to see the world with a broader vision and a higher angle, so as to communicate with people with different cultural orientations in a more flexible and efficient way [6]. Speculation is a kind of high-level psychological activity, which refers to the mental activity in which individuals make further solutions or decisions after analyzing and judging events, things, or phenomena according to certain standards. Its specific abilities include questioning reasoning, independent speculation, analysis and evaluation, etc.

Data mining (DM) [7] has been used in some theoretical studies in the area of education, primarily to examine how courses relate to one another, how to raise educational standards, how well students are prepared for their careers, and how different teachers with varying titles affect their students' learning. The main challenge in the application of the technology based on the DM analysis method in this paper is how to adopt the best DM algorithm to mine the data while simultaneously extracting the specific attributes that can reflect the system behavior and user behavior through the original knowledge data in accordance with each specific application demand. A DM algorithm that can be used to process a lot of students' information data is chosen, studied, and improved [8, 9] based on the characteristics of the behavior-related data of the students. Whether peer evaluation or student evaluation is used in the traditional teaching quality evaluation, the subjectivity and accuracy of the evaluation results cannot be avoided. In order to analyze teaching quality factors and uncover knowledge in a teaching-oriented data warehouse, the DM method is used in this paper.

The novelty of this study is that the DM method is combined with student achievement management and applied to real-world education, giving teachers a thorough understanding of students' overall learning situations, assisting schools in developing different reward and punishment schemes, and giving administrators more precise information resources for course offerings. Additionally, bettering teachers' instructional techniques can offer students more productive ways to learn. The aforementioned improvements can, in part, help to raise the management standard for college English speculative reading instruction as well as the calibre of that instruction.

## 2. Related Work

The competition between colleges and universities has grown over time as a result of the education system's ongoing reform and gradual development. The demand for managing student achievement has evolved from the initial simple input and recording operations to a situation where the hidden laws and values are mainly mined and the simple operations are supplemented at this time. The management of students' achievement in colleges and universities is progressively reaching a mature stage due to the intense demand for student achievement, and the strategy of mining the implicit information in student achievement data has emerged as the most significant area of research in these institutions [10].

Qiu digitally manages the personal information of all students in school, including personal bank cards, mobile phone numbers, public transportation IC cards used for going out, meal cards used in school daily life, and student insurance, and has established a relatively complete digital student behavior information management scheme. There are a lot of available data, which can be applied to data mining [11]. Zhao makes use of face-to-face teaching and autonomous learning mode, according to the data of students' feedback on learning English, teachers' interview with students' survey data, final evaluation, teachers' feedback, etc., to excavate students' autonomous learning [12]. Fei and Jiang think that the degree of students' development is determined only by one test result. This evaluation method masks the development process of teachers' teaching and students' learning, which not only fails to reflect the process and level of improvement of students' quality level but also makes it difficult to detect whether teachers have implemented quality education [13]. On the online English writing platform of Wang and Zhou, this paper uses the behavioral data of writing time, times of submission, changes in content, times of revision, etc., to excavate and analyze the factors that influence English writing and puts forward targeted solutions to improve English writing according to the influencing factors [14]. According to Liu, cross-cultural education and speculative reading instruction are both significant parts of contemporary college English speculative reading instruction. These components are beneficial to the development of students' cross-cultural communication ability and speculative ability and are supportive of students' adaptation to the development needs of the times and, ultimately, their realisation of their own value. Therefore, English teachers must focus on updating and optimizing the teaching content, vigorously carry out teaching and research activities, and innovate the teaching mode and concept in the practice of English speculative reading teaching in colleges and universities based on cross-cultural education. In order to encourage the orderly development of cross-cultural speculative teaching activities and to provide assurance for the development of English talents who can adapt to the changing nature of the world, colleges and universities should also strengthen the construction of their teaching staff [15]. According to Zhe, teacher preparation programs should be strengthened at colleges and universities. In order to improve the theoretical level and teaching abilities of all teachers, it is first important to strengthen the training and reeducation of current English teachers. This will allow for the further enrichment of teachers' English cultural knowledge reserves and cross-cultural speculative teaching abilities as well as the provision of assurance for effective and high-quality college English speculative reading teaching activities based on cross-cultural. Second, in order to improve the teaching level of English teachers overall through high-quality English education talents, we should actively introduce excellent English education talents, including foreign teachers with rich knowledge of British and American cultures. Excellent English education talents can introduce cutting-edge teaching concepts, teaching methods, teaching models, etc., in addition to the abundance of teaching resources, greatly enhancing the overall competency of teachers [16]. According to Chen, the core of cross-culturally based college English speculative reading instruction is teaching reform. If we want to effectively implement this in practice, we must focus on the growth of teaching and research activities that support innovation and the development of teaching mode and concept. To significantly increase students' cross-cultural communicative ability and critical thinking ability, it is first necessary to conduct a thorough analysis of cross-cultural speculative teaching and identify the cross-cultural educational concepts, teaching models, and teaching approaches that are consistent with college English speculative reading teaching [17]. Liu believes that language is the carrier of culture, and people cannot escape their own culture just like they cannot escape their own skin. In other words, when we are exposed to language, we are exposed to culture everywhere. As long as we pay enough attention to the “content” rather than the “form” of the text, we are learning culture “covertly.” Therefore, we can say that when a student is reading an original English text, he is experiencing a cross-cultural communication. Although it is only the communication between readers who do not meet each other, readers put themselves in the text during reading, on the one hand, accepting the meaning of the text, on the other hand, injecting their own knowledge into the text to expand the meaning of the text [18]. Examining students is one of the crucial ways, in the opinion of Xue, to assess a teacher's abilities, gauge their impact on students, and gauge the quality of their instruction. In order to implement high-quality education, it has become crucial to position exams accurately and use them properly. Students in their prime years and at the height of their intellectual development are in a unique position to both advance personally and significantly advance society. It is clear that one crucial aspect of educational reform is the way in which students' accomplishments are evaluated, and it is critical to find a quick solution to the examination system [19].

This paper finds that the current use of DM technology in college English speculative reading teaching primarily uses feedback data, such as test scores or questionnaires, to mine and analyze. This finding is based on the research of relevant scholars. How can the factors that are strongly related to test results according to learning path be mined and analyzed based on students' English training process or learning path data? With the help of portraits, this paper will mine and analyze the students' learning data from the college English speculative reading teaching and evaluation system. It will also use pertinent models to mine the test-related factors.

## 3. DM-Related Technologies

### 3.1. Data Preprocessing and Analysis

Many calculations must be performed on a relational database for the user's decision analysis to produce the desired results; however, the query results fall short of what the decision-makers require. The data in the data warehouse are typically multidimensional and arranged by topics, and they offer an OLAP query engine. Some analysis objects are known as metrics in the multidimensional data model, and the semantics of these metrics are dependent on the information of the dimensions that provide context semantics. The core of multidimensional data analysis algorithm research is how to effectively realise the aggregation operation in dimensions. This is because in the multidimensional data model of OLAP, the key operation is the aggregation operation of measurement attributes in some dimensions. Data is arranged into multiple dimensions in the multidimensional data model, and each dimension has multiple abstract layers determined by concept hierarchy [20]. Users can view and examine data in a variety of ways, thanks to this type of organization. In order for users to view the data in the data warehouse from different angles, sides, and levels and to fully understand the information connotation contained in the data, multidimensional analysis refers to various analysis actions such as slicing, cutting, rotating, and drilling on the data organized in multidimensional form. The mining process of database is shown in Figure 1.

The system indicates that DM objects are composed of databases, precise databases, data forms, or other information databases. The data query based on the semester grade table in the database contains many records, which cover the information content of all subjects of students in each semester. However, there are some defects in the design of student scholarship and scholarship information and competitive information. The items that these two tables have in common can be completely merged, and the data of these two tables can be merged. There are many similar data cleaning jobs, so the first step in the process of data cleaning is a major project. In this paper, the information gain rate is used instead of the information gain rate as the measure of attribute selection, and the definition of the evaluation function information gain rate is shown in

(1) $$\begin{array}{c} \text{Gain}\left(A\right)=\frac{G\left(A\right)}{E\left(A\right)}. \end{array}$$

In order to ensure the reasonable classification of samples, it is necessary to quantify the specific attributes of the selected samples. The quantified attributes are called sample indicators, and each sample has an indicator to indicate its behavior as shown in

(2) $$\begin{array}{c} u_{i}=\left(u_{i1},u_{i2},\cdots ,u_{\text{in}}\right),\;\left(i=1,2,\cdots ,n\right). \end{array}$$

In practical problems, different data usually have different dimensions and properties. In order to make the data with different dimensions meet the requirements of fuzzy DM algorithm, it is necessary to transform the original data. The steps of data standardization are shown in

(3) $$\begin{array}{c} u_{ik}=\left|\frac{u_{ik}-u_{k}}{S_{k}}\right|,\;\left(i=1,2,\cdots n\right),\left(k=1,2,3,4\right), \end{array}$$

(4) $$\begin{array}{c} u_{ik}=\frac{u_{1k}+u_{2k}+\cdots +u_{nk}}{\sum_{i=1}^{n}u_{ik}},\;\left(n=1,2,\cdots ,n\right). \end{array}$$

Although the change of standard deviation can eliminate the confusion caused by different dimensions between data, it cannot guarantee the transformed data, and it still needs to be transformed according to the extreme normalization formula, as shown in

(5) $$\begin{array}{c} u_{ik}=\frac{u_{ik}-u_{\min k}}{u_{\max k}},\;k=1,2,\cdots ,n. \end{array}$$

In the process of practical application, you can decide which algorithm to use according to different specific situations, as shown in (6) according to the traditional cluster analysis.

(6) $$\begin{array}{c} u_{ik}=\frac{u{\prime \prime }_{ik}-u{\prime \prime }_{\min k}}{u{\prime \prime }_{\max k}-u{\prime \prime }_{\min k}},\;k=1,2,\cdots ,n. \end{array}$$

The similarity coefficient method through translation range transformation is shown in

(7) $$\begin{array}{c} r_{ij}=\frac{\sum_{i=1}^{m}\left|x_{jk}-{\bar{x}}_{j}\right|\left|x_{jk}-{\bar{x}}_{i}\right|}{\sqrt{\sum_{j=1}^{m}\left(x_{jk}-{\bar{x}}_{j}\right)}}. \end{array}$$

The similarity coefficient can be obtained by exponential similarity coefficient method, in which the maximum-minimum method is shown in

(8) $$\begin{array}{c} r_{ij}=\frac{\sum_{j=1}^{m}\left(x_{ij}\Lambda x_{jk}\right)}{\sum_{i=1}^{m}\left(x_{ij}\nabla x_{jk}\right)}. \end{array}$$

The measure of similarity can also be determined by the corresponding measure of dissimilarity, as shown in

(9) $$\begin{array}{c} d\left(x_{j},x_{k}\right)=\left|x_{j1}-x_{k1}\right|+\left|x_{j2}-x_{k2}\right|+\cdots +\left|x_{jm}-x_{km}\right|, \end{array}$$

(10) $$\begin{array}{c} r_{ij}=\frac{\sum_{j=1}^{N}\left(a_{ij}\left(j\right)*r_{jk}\left(i\right)\right)}{\sum_{j=1}^{N}a_{jk}\left(x\right)}. \end{array}$$

The measure of dissimilarity is the same as the measure of similarity. The greater the dissimilarity, the smaller the similarity. On the contrary, the smaller the dissimilarity, the greater the similarity. For students at the whole school level, the amount of data is amazing. Therefore, in the actual work of selecting samples, undergraduate and junior college students have a huge amount of data, and there are many special places in graduate system and other undergraduate colleges. Because undergraduates are more representative and the data of students' behavior is huge, undergraduate students in colleges and universities are selected for data analysis. They are individual and special. In order not to affect the overall analysis effect in the overall situation, this paper adopts the data exclusion strategy for these students. From the point of view of accurate database, DM can be regarded as the advanced stage of online analytical processing, but the data analysis ability of DM based on advanced technologies of various data understanding far exceeds the online analytical processing function of accurate database, which mainly focuses on data aggregation.

### 3.2. Collection and Management of Data Warehouse

The majority of the data stored in data warehouses originates from the management information systems that colleges and universities currently have in place [21]. These systems have extremely valuable real-time and historical information because of the coexistence of various database management systems in colleges and universities, such as the educational administration management system and student management system. The collection of data warehouses is shown in Figure 2.

The student achievement analysis data warehouse contains a sizable amount of data and is focused on providing decision support for teaching management in colleges and universities. The data warehouse must be carefully designed to meet the demands of a rapid increase in data volume and no decrease in query performance due to factors like multidimensional structure, accurate requirements, and frequent updates [22]. After selecting the topic, it is necessary to thoroughly define the data that it contains as well as the connection between the fact table and the dimension table. It is essential to use English memorization as the cornerstone of the college English speculative reading curriculum so that students can read and learn English fluently on the assumption that they have mastered the necessary fundamental English knowledge. It is also important to focus on developing students' English analysis skills. This study proposes a DM-based approach for evaluating the effectiveness of college English speculative reading instruction and conducts an experimental verification. This paper uses DM technology to uncover the hidden, elusive, but valuable information of influencing factors of teaching quality from a large amount of data covering the procedure, conditions, and environment of college English teaching.

## 4. Analysis of the Teaching Quality of English Speculative Reading Based on Students' Behavior DM

### 4.1. Data Cleaning of Students' Behavior Characteristics

College English speculative reading teaching based on cross-cultural education has certain requirements for teaching content, and it is required to be related to social needs. At present, the content of English speculative reading teaching in colleges and universities is more about grammar, which is not conducive to the development of English speculative reading teaching based on cross-cultural education. First of all, the content of college English reading lacks cultural content. For a long time, the arrangement of English reading textbooks has been restricted by the traditional exam-oriented education, and more emphasis has been placed on English language knowledge, while the origin and development of English culture have not been introduced. If the teaching content of college English speculative reading fails to update with the times, it will affect the smooth development of English speculative reading teaching activities based on cross-cultural education. Secondly, the reading content lags behind and lacks advanced cultural content with the characteristics of the times. At present, the traditional textbook system is widely used in college English textbooks. Although some reforms have been made in the form, the failure to absorb the advanced cultural content with the characteristics of the times in English textbooks will also hinder the development of English speculative reading teaching. DM often depends on well-organized and preprocessed data sources, and the quality of data sources directly affects DM, so it is a very important stage in the process of data preparation. The data warehouse has various processing capabilities such as extracting data from various data, cleaning, and converting data, which just provides a good environment for DM to prepare data in the early stage.

As the main participants in the operation of colleges and universities, students are the main objects of teaching and learning, so it is particularly important to analyze their activities on campus. Mastering the knowledge and information of students' campus activities can better guide administrators to make the layout of the campus, arrange teaching activities reasonably, and optimize the management process. The research object in this paper is a group of university students majoring in English. The obvious progress of students' individual achievement (PMNP) is used as the objective evaluation index, and the factors influencing the obvious progress of students' individual achievement are examined using data on student behavior (DM). As shown in Table 1, statistics are created on the characteristics of various sample data in order to systematically observe the teaching factors that influence students' learning quality.

The clear progress rate of individual achievement serves as a measure of learning quality. The weight of the factors influencing PMNP can be determined using this decision tree. Because the DM algorithm automatically evaluates and categorises multivariate contingency tables based on the significance of the chi-square test, the closer it is to the decision root, the more significant the influencing factors are. Each node in the decision tree represents a distinct classification group determined by the DM algorithm, and the result data displays the impact of various factors on PMNP, as shown in Figure 3.

The construction of the teaching quality index system takes a new technical direction with the help of the DM-based teaching quality analysis method of college English speculative reading. This approach makes use of DM technology to sift through a sizable amount of data pertaining to the procedure, circumstances, and environment of college English teaching to uncover the hidden, elusive, but valuable information about factors that affect teaching quality. Each learning strategy has a unique impact, and students are free to choose the one that works best for them. As a result, in DM, the weighted sum of time is used as the learning time for each unit, and the students' final grades are used as the learning effect to engage in mining. The input data to be mined is obtained following the aforementioned data preprocessing procedure, as shown in Figure 4.

By analogy, until all the data records in the subset have the same values in the main attributes, or there are no attributes for division, complete student personal behavior data will be recursively formed. As the main body of English speculative reading teaching based on cross-cultural education, English teachers' ability and quality will affect the smooth development and effect of English speculative reading teaching. Therefore, it is very important to build a team of high-quality English teachers. However, at present, the construction level of English teachers in colleges and universities is low, and the overall quality of teachers is uneven, which is mainly reflected in the following aspects: first, teachers lack historical and cultural background and cultural teaching experience. Due to the lack of cultural knowledge and the lack of cross-cultural teaching experience, teachers can only simply introduce English culture in cross-cultural English speculative reading teaching but cannot carry out the specific teaching content in depth, which makes students only learn some simple English cultural knowledge, which directly restricts the improvement of students' English cultural literacy. Secondly, teachers' mastery of English knowledge is not solid, and they are seriously short of advanced educational concepts. More importantly, English teachers are not aware of the importance of English speculative reading teaching based on cross-cultural education. To some extent, these results show that our extracted behavior characteristics have certain effect on the prediction of students' academic performance. The comparison of evaluation indexes of each model in this paper is shown in Figure 5.

The structure of this paper is adaptable enough for early warning because of the variety of students' activities and the limitations of data collection techniques. Additionally, using the parameters of the model, it is possible to quantitatively assess the relationship between daily behavior and academic performance. In order for students to read and learn English fluently on the assumption that they have mastered relevant basic English knowledge, it is important to prioritise the development of students' English analysis skills. This is especially important when teaching college students to read speculatively in English. We can reduce the teaching content of superficial English dialogue and increase the training content of argumentation and analysis of specific problems that concentrate on the analysis of English thinking. We can also appropriately increase the training of English argumentation and writing in classroom design. In cross-cultural education, the development of speculative reading instruction in English has raised the bar for the teaching approach. Numerous issues with the teaching approach exist in the classroom and directly impede the growth of the teaching of speculative reading in English. The traditional teaching approach used in English reading instruction does not adapt to the times, leaving it unable to meet the demands of cross-cultural college English speculative reading instruction. It becomes easier to optimize and innovate the teaching mode, but it is more difficult to carry out targeted and in-depth teaching and research work in accordance with the requirements of English speculative reading teaching based on cross-cultural education. This limits the effective development of English speculative reading teaching activities.

### 4.2. Data Analysis of Students' Achievement Based on Data Warehouse

The key to whether teaching activities are successful or unsuccessful is determining the teaching objectives. Teachers should focus on developing students' critical thinking and cross-cultural competence while also striking a balance between teaching content and the English language and ensuring that it is used accurately and fluently. Cross-cultural speculative reading teaching must firmly grasp the three training objectives of language ability, cross-cultural ability, and speculative ability, so that they can develop in a balanced way and promote each other. According to the idea of multidimensional analysis of users, this paper looks at the distribution of students' public course scores in all academic years from the perspective of class and according to the course type, which, respectively, contains two dimensions, one is the course information dimension, and the other is the course type. The second is class name dimension, which takes the class as granularity and the measured value as average score. Drag the class name dimension into the row of the table model, drag the course information dimension into the column of the table model, and finally drag the measured student average score into the data area of the table model, as shown in Figure 6.

For student management workers, students in different classes, different grades, and different majors can be investigated and analyzed, and the characteristics of the classes with good overall English scores can be analyzed, while the reasons can be analyzed for the classes with higher professional scores but average or even poor English scores when entering the school. Bit table is a set of integers, each bit of which represents an item. In this fast frequent itemset mining, bit table is used to compress candidate set and database. For candidate set compression, if the candidate set contains items, the position of items in the table is 1; otherwise, it is 0. For database compression, bit table can be used directly, as shown in Table 2.

Through the observation and analysis of the above tables, it is found that there are a lot of redundant information. For example, the student table itself contains detailed information of students, including all kinds of information such as classes. However, there are the same data information in the scholarship table. This redundant data information is worthless in data analysis but increases the burden of the analysis system. The data in the data tables involved in the system are subjected to rule reduction, and some attributes are selected for integration operation to generate new attributes. Finally, the conclusion is that it is more conducive to the data analysis of the whole information table. The student data information in the system comes from different data sources. Integrating the data in these data sources to form a unified data set provides convenient conditions for the behavior analysis of the student data in the system. In this paper, the commonly used clustering analysis algorithms are analyzed and studied by using the MATLAB software, and the analysis results of the algorithms are obtained from different angles and compared. The MATLAB experimental output results are shown in Figure 7.

Through the relevant research and discussion on the principles of the above four algorithms and the process of clustering algorithm, this paper chooses MATLAB program to design and implement the programming operation. The number of wrong samples is the sum of all the wrong samples generated by each clustering method in the clustering process. Among them, the average prediction accuracy of DM algorithm is 0.86, while the three algorithms are 0.71, 0.75, and 0.73, respectively, which shows that the DM algorithm in this paper has a better effect on predicting students' English scores. In the teaching activities of college English speculative reading, imitation learning and observation learning are a primary behavior mode, which mainly follows the example. Teachers should guide students to study and think independently in imitation learning and observation learning; give full play to students' subjective initiative and creativity; make a deep summary, induction, and innovation of English knowledge; and carry out creative learning of English knowledge based on their own understanding. In the teaching of observing and guiding innovation in English, different ways can be introduced, such as sitcom performance and microclassroom presentation, to guide students to interact, communicate, and talk in English reading, supplemented by reflection and evaluation teaching, so as to cultivate students' thinking ability.

## 5. Conclusions

Carrying out cross-cultural English speculative reading teaching is essentially a reform of education and teaching. To do this teaching effectively, we must carry out in-depth teaching and research activities. First, we must change the teaching methods and actively carry out independent inquiry teaching, which can effectively stimulate students' learning desire and enthusiasm. In traditional teaching, teachers are in the dominant position, and the classroom is filled by teachers and passively accepted by students, which is not conducive to stimulating students' learning enthusiasm. To carry out self-inquiry teaching is to return the subject status to the students, to enable them to learn independently under the guidance and maintenance of teachers, and to cultivate their self-learning ability. Second, we should vigorously carry out cross-cultural education and teaching research, timely determine the ideas, modes, and methods of cross-cultural education suitable for the actual situation of our unit, and cultivate and enhance students' cross-cultural communication ability. Third, we should carry out in-depth research on speculative reading teaching, adopt diversified teaching modes and methods in combination with the teaching practice of our unit, and constantly improve students' cross-cultural mentality and speculative ability. Fourthly, we should boldly introduce the teaching ideas and methods of multimedia education and promote the in-depth reform of teaching ideas and teaching models. The experimental data sources involved in the prediction platform of students' behavior characteristics set up in this paper are limited, and the evaluation indexes and research results of students' behavior characteristics cannot fully reflect students' learning and living behaviors in school. Therefore, in the follow-up research, it is necessary to improve the data sources, make the evaluation indexes of students' behavior more detailed, and make the research results more accurate and comprehensive. The follow-up research can carry out real-time data preprocessing and mining analysis by establishing a distributed processing platform for real-time streaming data.

## Figures and Tables

**Figure 1:** DM process.

**Figure 2:** Data warehouse architecture.

**Figure 3:** Statistical data indicators of nodes.

**Figure 4:** Preprocessing data.

**Figure 5:** Comparison between single-task model and multitask model.

**Figure 6:** Average English scores in colleges and universities of various majors.

**Figure 7:** Comparative experimental results of algorithms.

**Table 1:** Sample characteristics.

Attribute	Attribute value	Proportion of sample
Students' gender	Man	57.3%
	Woman	42.7%
Teaching means	Multimedia teaching means are abundant	65.9%
	Little or insufficient multimedia teaching	34.1%
Learning purpose	Pass the exam	33.2%
	Interest	52.4%
	Looking for a job or going abroad	14.3%
Overall evaluation of students' teachers	Excellent	56.5%
	Good	37.3%
	Medium or poor	6.2%
Evaluation of students' difficulty in examination	Relatively difficult	24.9%
	Proper	57.8%
	Pianyi	17.3%
Students' evaluation of teaching materials	Good	39.8%
	Common	45.2%
	Be poor	15.0%

**Table 2:** Compression bit table of student behavior data.

TID	Item 1	Item 2	Item 3	Item 4	Item 5
1	1	0	0	0	1
2	1	0	1	1	1
3	0	0	1	0	0
4	1	1	0	1	1
Bit table	16	12	18	17	14

## Data Availability

The data used to support the findings of this study are available from the corresponding author upon request.
